The article "Gene-Expression Changes in Cerium Chloride-Induced Injury of Mouse Hippocampus" was retracted in 2024. Reasons: plagiarized text; duplicated images; duplicated data; duplicated text.

# Gene-Expression Changes in Cerium Chloride-Induced Injury of Mouse Hippocampus

**DOI:** 10.1371/journal.pone.0060092

**Published:** 2013-04-03

**Authors:** Zhe Cheng, Haiquan Zhao, Yuguan Ze, Junju Su, Bing Li, Lei Sheng, Liyuan Zhu, Ning Guan, Suxin Gui, Xuezi Sang, Xiaoyang Zhao, Qingqing Sun, Ling Wang, Jie Cheng, Renping Hu, Fashui Hong

**Affiliations:** 1 Medical College of Soochow University, Suzhou, P. R. China; 2 College of Life Sciences, Anhui Agriculture University, Hefei, P. R. China; Indian Institute of Toxicology Research, India

## Abstract

Cerium is widely used in many aspects of modern society, including agriculture, industry and medicine. It has been demonstrated to enter the ecological environment, is then transferred to humans through food chains, and causes toxic actions in several organs including the brain of animals. However, the neurotoxic molecular mechanisms are not clearly understood. In this study, mice were exposed to 0.5, 1, and 2 mg/kg BW cerium chloride (CeCl_3_) for 90 consecutive days, and their learning and memory ability as well as hippocampal gene expression profile were investigated. Our findings suggested that exposure to CeCl_3_ led to hippocampal lesions, apoptosis, oxidative stress and impairment of spatial recognition memory. Furthermore, microarray data showed marked alterations in the expression of 154 genes involved in learning and memory, immunity and inflammation, signal transduction, apoptosis and response to stress in the 2 mg/kg CeCl_3_ exposed hippocampi. Specifically, the significant up-regulation of Axud1, Cdc37, and Ube2v1 caused severe apoptosis, and great suppression of Adcy8, Fos, and Slc5a7 expression led to impairment of mouse cognitive ability. Therefore, Axud1, Cdc37, Ube2v1, Adcy8, Fos, and Slc5a7 may be potential biomarkers of hippocampal toxicity caused by CeCl_3_ exposure.

## Introduction

Due to their diverse physical, chemical, and biological effects, lanthanides (Ln) have been increasingly used in many aspects of modern society, including agriculture (fertilizers and animal breeding), industry (color TV, photographic cameras, semiconductors, movie films) [1], [2] and in medicine as anticancer, anti-inflammatory, and antiviral agents [3]. Recently, numerous studies have also suggested that CeCl_3_ and cerium oxide nanoparticles have potential positive effects on fibroblast and osteoblast proliferation and differentiation [4], cutaneous wound healing [5], and downregulation of tumor growth and invasion [6]. Due to the widespread application of Ln,they inevitably enter the ecological environment and are then transferred to humans through food chains [7]. It was reported that the average intake of Ln was about 1.75–2.25 mg/day in China; and may be 5–10 times higher in the Ln ore district [8]. Therefore, the toxicological effects of Ln in humans are a concern.

Cerium, is a typical rare earth element, and is one of the most frequently used elements in Ln. It was found that high doses of Ce^3+^ induced liver and kidney lesions and induced enzyme metabolic disorders in animals [9], [10]. Li et al. found increases in creatinine, ketone bodies, succinate, lactate, and various amino acids in the serum of rats acutely exposed to Ce^3+^ for 48 h, as well as a reduction in serum dextrose [11]. These authors suggested that Ce^3+^ at high doses damaged a specific region of the liver. A recent study showed that exposure to Ce^3+^ damaged the spleen [12], [13], lung [14]), and liver [15]–[17] of mice. In addition, La^3+^, Ce^3+^ and Nd^3+^ were demonstrated to result in brain injuries in mice [18]–[20]. In the early 1990s, it was reported that the mean memory and intelligence quotient (IQ) value in children aged 6 to 9 years in rare-earth polluted areas were significantly lower than those in non-polluted areas [21]. Feng et al. suggested that La^3+^ could affect learning ability, which may be ascribed to disturbance in the homeostasis of trace elements, enzymes and neurotransmitter systems in the rat brain [22]. Other studies showed that short-term exposure to La^3+^- and Ce^3+^ significantly decreased total antioxidant level and the activities of Na^+^, K^+^-ATPase, and increased the activities of acetylcholinesterase in rat brain [23. 24]. Our previous study suggested that cerium was significantly accumulated in the mouse hippocampus, and in turn caused hippocampal apoptosis and impairment of spatial recognition memory in mice exposed to CeCl_3_ for 60 consecutive days [20]. These data indicated that Ln affects the central nervous system (CNS), especially cognitive ability. Although the above-mentioned studies clarified the neurotoxic effects of Ln, further studies are needed to elucidate the synergistic molecular mechanisms of multiple genes activated by Ln-induced nuerotoxicity in animals and humans. We speculate that CeCl_3_-induced CNS damages in mice may have special biomarkers of nuerotoxicity.

Microarray technology has been used as a screening tool for the identification of molecular mechanisms involved in toxicity [25]. Large-scale gene expression analysis provides a logical approach for researchers to identify those genes and their products which are involved in conferring resistance or susceptibility to toxic substances. In the present study, we aimed to investigate hippocampal dysfunction caused by CeCl_3_ exposure and alterations in the gene expression profile in mouse hippocampus using microarray analysis. The data on gene expression profiling showed significant changes in genes involved in learning and memory, immunity and inflammation, signal transduction, apoptosis, and response to stress in the CeCl_3_ exposed hippocampi. Our findings may provide a reference for future mechanistic studies on the effects of Ln on brain tissues in animals or humans.

## Materials and Methods

CeCl_3_ was purchased from Shanghai Chem. Co. (China) and was of analytical grade (99.99%).

### Ethics Statement

All experiments were conducted during the light phase, were approved by the Animal Experimental Committee of Soochow University (Grant 2111270) and were in accordance with the National Institutes of Health Guidelines for the Care and Use of Laboratory Animals (NIH Guidelines).

### Animals and Treatment

Male CD-1 (ICR) mice (18±2 g, 4 weeks old) were purchased from the Animal Center of Soochow University (Suzhou, China), and were housed in polypropylene cages with corncob bedding in a controlled-environment animal room (temperature, 24±1°C; relative humidity, 60±10%; photoperiod, 12 h light/dark cycle).

Three hundred animals were randomly divided into four groups (75 mice/group): control group (treated with purified water) and three experimental groups (treated with 0.5, 1, and 2 mg/kg body weight [BW] CeCl_3,_ respectively). With regard to the dose selection in this study, we identified the average intake of Ln (1.75–2.25 mg/day) in humans [8]. The mice were weighed and the CeCl_3_ solutions were administered intragastrically every day for 90 days. Symptoms and mortality were carefully observed and recorded every day for 90 days (death not observed).

### Behavioral Experiment

Following 90 days of CeCl_3_ administration, the acquisition of spatial recognition memory in mice (N = 20) was determined using the Y-maze test. In order to avoid any stress-related interference with the learning procedure, mice were not handled by the experimenter, but were allowed to voluntarily enter the maze. To assess spatial recognition memory, the Y-maze test consisted of two trials separated by an intertrial interval (ITI). The Y-maze was made of green–blue painted timber and consisted of three arms with an angle of 120° between each two arms. Each arm was 8 cm × 30 cm × 15 cm (width × length × height). The three identical arms were randomly designated: Start arm, in which the mouse started to explore (always open), Novel arm, which was blocked during the 1^st^ trial, but open during the 2^nd^ trial, and the Other arm (always open).

The maze was placed in a sound attenuated room with low illumination. The floor of the maze was covered with sawdust, which was mixed after each individual trial in order to eliminate olfactory stimuli. Visual cues were placed on the walls of the maze, and the observer was always in the same position at least 3 m from the maze.

The Y-maze test consisted of two trials separated by an ITI to assess spatial recognition memory. The first trial was of 10-min duration and allowed the mouse to explore only two arms (Start arm and Other arm) of the maze, with the third arm (Novel arm) being blocked. After a 1 h ITI, the second trial (retention) was conducted, during which all three arms were accessible and novelty vs. familiarity was analyzed by comparing behavior in all three arms. For the second trial, the mouse was placed back into the maze in the same starting arm, with free access to all three arms for 5 min. By using a ceiling-mounted CCD camera, all trials were recorded on a VCR. Video recordings were later analyzed and the number of entries and time spent in each arm were analyzed. Data were also expressed as percentage of total time and distance spent in arms every 30 s and during the total 5 min period [26]. In the second trial, we also assessed which of the arms was entered first as another way of recognizing the Novel arm–discrimination memory. Because retention in the Y-maze test does not last longer than a few hours, this task can be assessed three times in the same animal [27]. All mice were therefore tested in the Y-maze three times using a 1 h ITI. There was no arm difference in animals treated with CeCl_3,_ but when compared to the control, animals in this group spent less time in the Novel arm indicating that animals in this group failed to recognize the Novel arm after the 1 h ITI.

To measure spatial recognition memory, the number of entries and time spent in each arm of the maze by each mouse was recorded and novelty versus familiarity was analyzed by comparing behavior in all three arms. The number of arms visited was taken as an indicator of locomotor and exploratory activity.

### Preparation of Hippocampus

After the behavioral experiments, all animals were first weighed and then sacrificed after being anesthetized by ether. The brains were quickly removed and placed in ice-cold, and the hippocampi were dissected and frozen at −80°C.

After weighing the body and brains, the coefficient of brain mass to BW was calculated as the ratio of brain (wet weight, mg) to BW (g).

### Histopathological Examination of the Hippocampus

For pathologic studies, all histopathologic examinations were performed using standard laboratory procedures. The hippocampi were embedded in paraffin blocks, then sliced (5 µm thickness) and placed onto glass slides. After hematoxylin–eosin staining, the stained sections were evaluated by a histopathologist unaware of the treatments, using an optical microscope (Nikon U-III Multi-point Sensor System, Japan).

### Observation of Hippocampus Ultrastructure

Hippocampi were fixed in a fresh solution of 0.1 M sodium cacodylate buffer containing 2.5% glutaraldehyde and 2% formaldehyde followed by a 2 h fixation period at 4°C with 1% osmium tetroxide in 50 mM sodium cacodylate (pH 7.2–7.4). Staining was performed overnight with 0.5% aqueous uranyl acetate. The specimens were dehydrated in a graded series of ethanol (75, 85, 95, and 100%), and embedded in Epon 812. Ultrathin sections were obtained, contrasted with uranyl acetate and lead citrate, and observed with a HITACHI H600 Transmission Electron Microscope (TEM) (HITACHI Co., Japan). Hippocampal apoptosis was determined based on the changes in nuclear morphology (e.g., chromatin condensation and fragmentation).

### Analysis of Hippocampal Cerium Content

The frozen hippocampal tissues were thawed and ∼ 0.1 g samples were weighed, digested, and analyzed for cerium content. Briefly, prior to elemental analysis, the lung tissues were digested overnight with nitric acid (ultrapure grade). After adding 0.5 mL of H_2_O_2_, the mixed solutions were incubated at 160°C in high-pressure reaction containers in an oven until the samples were completely digested. The solutions were then incubated at 120°C to remove any remaining nitric acid until the solutions were colorless and clear. Finally, the remaining solutions were diluted to 3 mL with 2% nitric acid. Inductively coupled plasma-mass spectrometry (Thermo Elemental X7; Thermo Electron Co., Waltham, MA, USA) was used to determine the cerium concentration in the samples. Indium (20 ng/mL) was chosen as an internal standard element. The detection limitation of cerium was 0.074 ng/mL and data are expressed as ng/g of fresh tissue.

### Oxidative Stress Assay

Reactive oxygen species (ROS) (O_2_ **^−^** and H_2_O_2_) production and levels of malondialdehyde (MDA), protein carbonyl (PC), and 8-hydroxy deoxyguanosine (8-OHdG) in the hippocampal tissues were assayed using commercial enzyme-linked immunosorbent assay kits (Nanjing Jiancheng Bioengineering Institute, Jiangsu, China) according to the manufacturer’s instructions.

### Microarray and Data Assay

Gene expression profiles in hippocampal tissue isolated from 5 mice in the control and CeCl_3_-treated groups were compared by microarray analysis using Illumina BeadChip purchased from Illumina, Inc. (San Diego, CA, USA). Total RNA was isolated using the Ambion Illumina RNA Amplification Kit (cat no. 1755) according to the manufacturer’s protocol, and stored at −80°C. RNA amplification is the standard method for preparing RNA samples for array analysis [28]. Total RNA was then submitted to the Biostar Genechip Inc. (Shanghai, China) where RNA quality was analyzed using a BioAnalyzer, and cRNA was generated and labeled using the one-cycle target labeling method. cRNA from each mouse was hybridized for 18 h at 55°C on Illumina Human HT-12 v 3.0 BeadChips, containing 45, 200 probes (Illumina, Inc., San Diego, CA, USA), according to the manufacturer’s protocol and subsequently scanned with the Illumina BeadArray Reader 500. This program identifies differentially expressed genes and establishes the biological significance based on the Gene Ontology Consortium database (http://www.geneontology.org/GO.doc.html, _GSE44906_). Data analyses were performed with GenomeStudio software version 2009 (Illumina Inc., San Diego, CA, USA), by comparing all values obtained at each time point against the 0 h values. Data were normalized with the quantile normalization algorithm, and genes were considered as detected if the detection p-value was lower than 0.05. Statistical significance was calculated using the Illumina DiffScore, a proprietary algorithm that uses the bead standard deviation to build an error model. Only genes with a DiffScore ≤-13 and ≥13, corresponding to a p-value of 0.05, were considered statistically significant(You et al., 2010; Grober Oli et al., 2011).

### Quantitative Real-time PCR (qRT-PCR)

Expression levels of Adcy8, Axud1, Cdc37, Fos, Slc5a7, and Ube2v1 mRNA in mouse hippocampal tissues were determined using real-time quantitative reverse transcriptase polymerase chain reaction (qRT-PCR) [29]. Synthesized complimentary DNA was generated by qRT-PCR with primers designed with Primer Express Software (Applied Biosystems, Foster City, CA, USA) according to the software guidelines, and PCR primer sequences are listed in Table 1.

**Table 1:** Real time PCR primer pairs. PCR primers used in the gene expression analysis.

Gene name	Description	Primer sequence	Primer size (bp)
**Refer-actin**	mactin-F	5′-GAGACCTTCAACACCCCAGC-3′	
	mactin-R	5′-ATGTCACGCACGATTTCCC-3′	263
**Slc5a7**	mSlc5a7-F	5′-TTCCAGATTCAGGCAGTAGACG-3′	
	mSlc5a7-R	5′-GGGAGGGAAACTCCTATCTTGT-3′	125
**Fos**	mFos-F	5′-TGTACTGTAGTCCTTCAGCGTCA-3′	
	mFos1-R	5′-TGTCAGAACATTCAGACCACCTC-3′	82
**Adcy8**	mAdcy8-F	5′-GGAGAAACAGACTTCCTGGGTACAA-3′	
	mAdcy8-R	5′-CATTGTGCTCCCTTAACTCCTTCATTTC-3′	175
**Axud1**	mAxud1-F	5′-CGCCCTTCATTAGCTGATGTT-3′	
	mAxud1-R	5′-CAGAGCCTGCGTTTCTTGG-3′	117
**Ube2v1**	mUbe2v1-F	5′-GATAGAGTGTGGGCCTAAGTACC-3′	
	mUbe2v1-R	5′-TGAGCAGTTCGAATGGAGTG-3′	120
**Cdc37**	mCdc37-F	5′-CTGTCAGACAACGTCCACCTG-3′	
	mCac37-R	5′-CGAAGCACTTCTGGAGTTCCT-3′	88

### ELISA Assay

To determine Adcy8, Axud1, Cdc37, Fos, Slc5a7, and Ube2v1 levels in mouse hippocampal tissues, Enzyme Linked Immunosorbent Assay (ELISA) was performed using commercial kits that were selective for each respective protein (R&D Systems, USA), following the manufacturer’s instructions. The absorbance was measured on a microplate reader at 450 nm (Varioskan Flash, Thermo Electron, Finland), and the concentrations of Adcy8, Axud1, Cdc37, Fos, Slc5a7, and Ube2v1 were calculated from a standard curve for each sample.

### Statistical Analysis

All results are expressed as means ± standard error of the mean(SEM). The significant differences were examined by unpaired Student’s t-test using SPSS 19 software (USA). A p-value <0.05 was considered as statistically significant.

## Results

### Spatial Recognition Memory

The effects of CeCl_3_ on the spatial recognition memory of mice are presented in Fig. 1. From this figure it can be seen that the percentage duration in the novel arm in control mice was significantly higher than that in the start and other arms throughout the experiment, while the percentage duration in the novel arm in 0.5, 1 and 2 mg/kg CeCl_3_ -treated mice was lower than that of control mice (P<0.05), respectively. These results suggest that exposure to low-dose CeCl_3_ for a long period impaired the spatial recognition memory of mice. This might be related to brain injury, which was confirmed by morphological examination.

**Figure 1:** Effect of CeCl_3_ on spatial recognition memory in mice in the Y-maze test following intragastric administration of CeCl_3_ for 90 consecutive days. Different letters indicate significant differences between groups (p<0.05). Values represent means ± SEM (N = 20).

### Locomotor Activity

The effect of CeCl_3_ on arm visits is presented in Fig. 2. The results indicated that CeCl_3_ dose-dependently decreased the number of arm entries compared to the control. Measurement of total number of arm entries during the second trial revealed a significant difference between the three arms in each group after the 1 h ITI.

**Figure 2:** Effects of acute CeCl_3_ locomotor activity of mice in the Y-maze test following intragastric administration of CeCl_3_ for 90 consecutive days. Different letters indicate significant differences between groups (p<0.05). Values represent means ± SEM (N = 20).

### BW, Relative Brain Weight, and Cerium Accumulation

BW, relative brain weight and cerium accumulation in mice are listed in Table 2. As shown, an increase in CeCl_3_ dose led to a gradual decrease in BW, and relative brain weight, whereas cerium content was significantly increased (*p*<0.05), indicating growth inhibition and brain damage in mice. These findings were confirmed by subsequent hippocampus histological and ultrastructural observations and oxidative stress assays.

**Table 2:** Body weight, relative weight of brain and cerium accumulation in mouse hippocampus after intragastric administration of CeCl_3_ for 90 consecutive days.

Index	CeCl_3_ (mg/kg BW)			
	0	0.5	1	2
**Net increase of body weight (g)**	23±1.15a	19±0.95b	14±0.70c	10±0.50d
**Relative weight of brain (mg/g)**	16.08±0.80a	14.59±0.73a	11.37±0.57b	8.98±0.45c
***Cerium content*** ***(ng/g tissue)***	Not detected	150±7.50a	288±14.40b	609±30.45c

Different letters indicate significant differences between groups (p<0.05). Values represent means ± SEM (N = 10).

### Histopathological Evaluation

The histopathological changes in mouse hippocampus are presented in Fig. 3. It can be seen that exposure to CeCl_3_ resulted in abnormal pathological changes in the hippocampi when compared with the control group, including overproliferation of all glial cells, tissue necrosis and bleeding, indicating that the CNS was injured by exposure to CeCl_3_.

**Figure 3:** Histopathology of hippocampi in mice caused by intragastric administration of CeCl_3_ for 90 consecutive days (N = 5). (a) Control group; (b) 0.5 mg/kg CeCl_3_ group indicates significant proliferation of all glial cells; (c) 1 mg/kg CeCl_3_ group indicates significant proliferation of all glial cells and tissue necrosis; (d) 2 mg/kg CeCl_3_ group indicates significant proliferation of all glial cells, tissue necrosis and bleeding.

### Hippocampal Cell Ultrastructure

The changes in hippocampal cell ultrastructure in mice are shown in Fig. 4. It was observed that the neurons in the control group contained elliptical nuclei with homogeneous chromatin. However, the hippocampal cell ultrastructure in the CeCl_3_-treated mice showed typical apoptosis, including irregularity of nuclear membrane, shrinkage of the nucleus, chromatin marginalization, mitochondrial swelling and ectatic endoplasmic reticulum. These results suggested that exposure to low doses of CeCl_3_ caused hippocampal apoptosis, which might affect spatial recognition memory in mice.

**Figure 4:** Ultrastructure of hippocampal cells in mice caused by intragastric administration of CeCl_3_ for 90 consecutive days (N = 5). (a) Control group indicates nucleus with homogeneous chromatin; (b) 0.5 mg/kg CeCl_3_ group indicates irregularity of nuclear membrane, shrinkage of nucleus, chromatin marginalization, and mitochondrial swelling; (c) 1 mg/kg CeCl_3_ group indicates irregularity of nuclear membrane, severe shrinkage of nucleus, chromatin marginalization, and mitochondrial swelling; (c) 2 mg/kg CeCl_3_ group indicates significant irregularity of nuclear membrane, severe shrinkage of nucleus, chromatin marginalization, mitochondrial swelling, and ectatic endoplasmic reticulum.

### Analysis of Oxidative Stress

To further confirm hippocampal apoptosis, we detected ROS generation rate, and levels of lipids, proteins, and DNA peroxidation. The effects of CeCl_3_ on the production of O_2_^−^ and H_2_O_2_ in mouse hippocampal tissues are shown in Table 3. With increased CeCl_3_ dose, the rate of ROS generation in the CeCl_3_-exposed groups was significantly elevated (*p*<0.05), suggesting that exposure to CeCl_3_ accelerated ROS production in the hippocampal tissues. As shown in Table 3, levels of MDA, PC, and 8-OHdG in the hippocampal tissues from the CeCl_3_-exposed groups were markedly elevated (*p*<0.05), suggesting that CeCl_3_–induced ROS accumulation led to lipid, protein, and DNA peroxidation.

**Table 3:** Oxidative stress in mouse hippocampus after intragastric administration of CeCl_3_ for 90 consecutive days.

Oxidative stress	CeCl_3_ (mg/kg BW)			
	0	0.5	1	2
**O_2_^−^ (nmol/mg** **prot. min)**	31.05±1.55	40.86±2.04	52.89±2.64	67.50±3.38
**H_2_O_2_ (nmol/mg prot. min)**	58.05±2.90	82.64±4.13	106.60±5.33	148.50±7.42
**MDA (µmol/mg prot)**	1.46±0.07	2.15±0.11	3.90±0.19	6.95±0.35
**Carbonyl (µmol/** **mg prot)**	0.73±0.04	1.32±0.07	2.50±0.12	4.10±0.21
***8-OHdG (mg/g tissue)***	0.57±0.03	3.05±0.15	5.74±0.29	9.61±0.48

Different letters indicate significant differences between groups (p<0.05). Values represent means ± SEM (N = 5).

### Gene Expression Profile

Treatment with 2 mg/kg BW of CeCl_3_ resulted in the most severe hippocampal damage and these tissues were used to determine gene expression profiles to further explore the mechanisms of hippocampal damage induced by CeCl_3_. The results showed that 244 genes were obviously altered in brain tissue following exposure to CeCl_3_ compared with the control group. Of the genes altered, 194 genes were up-regulated and 50 genes were down-regulated. Alterations in the known gene expression profile induced by exposure to CeCl_3_ for 90 consecutive days are shown in Table S1. The gene expression profile of the hippocampal tissues from the CeCl_3_-treated mice was classified using the ontology-driven clustering algorithm included with the PANTHER Gene Expression Analysis Software (www.pantherdb.org/), which suggested that 154 genes in the gene expression profile were divided into 10 cluster categories including learning and memory, transcription, signal transduction, cell structure and cytoskeleton, growth and development, metabolism, immunity and inflammation, apoptosis, response to stress and translation (Fig. 5), and the function of 90 genes was unknown.

**Figure 5:** Gene expression changes in mouse hippocampus following intragastric administration of 2 mg/kg BW CeCl_3_ for 90 consecutive days. Selection of over-represented biological categories that include differentially expressed genes. Rows represent gene categories and the percentage of the genes included in each category to the total number of differentially expressed genes, and the number of genes is indicated on the right side of each bar.

### qRT-PCR

To verify the accuracy of the microarray analysis, six genes that demonstrated significantly different expression patterns were further evaluated by qRT-PCR due to their association with learning and memory, apoptosis and oxidative stress. These 3 genes including Axud1, Cdc37, and Ube2v1 were up-regulated, whereas 3 genes including Adcy8, Fos, and Slc5a7 were down-regulated (Table 4). The qRT-PCR analysis of all 6 genes displayed expression patterns comparable with the microarray data (i.e., either up- or down-regulation; Table S1).

**Table 4:** RT-PCR validation of selected genes from Microarray Data.

Function	Gene	△△Ct	Fold	Microarray data (Fold)
**learning and memory**	***Slc5a7***	0.71±0.04	0.61±0.03a	0.52±0.03a
	***Fos***	1.82±0.09	0.28±0.01a	0.43±0.02b
	***Adcy8***	0.40±0.02	0.76±0.04a	0.54±0.03b
**Apoptosis**	***Axud1***	−3.40±0.17	10.59±0.53a	14.13±0.71b
	***Ube2v1***	−1.77±0.09	3.40±0.17a	2.59±0.13b
	***Cdc37***	−1.33±0.07	2.51±0.13a	26.25±1.31b

Different letters indicate significant differences between groups (p<0.05). Values represent means ± SEM (N = 5).

### ELISA

In order to further confirm expression of Adcy8, Axud1, Cdc37, Fos, Slc5a7, and Ube2v1 in hippocampal tissues, their protein levels were measured by ELISA. The expression levels of Axud1, Cdc37, and Ube2v1 proteins in hippocampus were gradually elevated following exposure to 2 mg/kg CeCl_3_, whereas the levels of Adcy8, Fos, and Slc5a7 in CeCl_3_-exposed mice were lower than those in unexposed mice (Fig. 6).

**Figure 6:** Effect of CeCl_3_ on the levels of protein expression in mouse **hippocampus following intragastric administration of CeCl_3_ for 90 consecutive days.** Different letters indicate significant differences between groups (p<0.05). Values represent means ± SEM (N = 5).

## Discussion

The results of this study indicated that exposure to low dose CeCl_3_ for 90 days resulted in decreases in spatial recognition memory (Fig. 1). According to Dellu et al., the two-trial Y-maze task is a specific and sensitive test of spatial recognition memory in rodents [27]. Our data supported this view by showing that there were always significant arm effects on percentage measures of total duration of visits and number of visits during the retention test. Following exposure to increased doses of CeCl_3_, the time spent in the unfamiliar novel arm, and or the frequency with which mice entered this arm, were not statistically different from the familiar start and other arms after the 1 h ITI. However, in unexposed mice, the time spent in the unfamiliar novel arm, and or the frequency with which mice entered these arms, were higher than those for the familiar start and other arms (Fig. 1). This suggested that mice were highly sensitive to their spatial and contextual environment. Moreover, our data were consistent with previous findings in CD1 mice which demonstrated a very high level of novelty exploration [27]. In the retention test, mice had to make a choice between the novel arm (unfamiliar) and the other arm (familiar) when they were released from the start arm in the Y-maze. Mice exposed to CeCl_3_ showed a lower score in discrimination memory than unexposed mice. Our findings demonstrated that CeCl_3_ may impair spatial recognition memory in mice in the Y-maze. Locomotor activity is a function of the level of excitability of the central nervous system [30]. We found that CeCl_3_ reduced locomotor activity in mice. Furthermore, in the CeCl_3_-exposed mice, the reduction in learning and memory was coupled with a reduction in brain indices, cerium accumulation (Table 2), severe hippocampal lesions (Figs. 2, 3) as well as oxidative stress (Table 3). These injuries may be associated with alterations in gene expression in the hippocampus. To identify the molecular mechanisms of multiple genes working together following exposure to CeCl_3_, microarray assays of hippocampal RNA were performed to establish a global gene expression profile. These assays suggested (Table S1) that the expression levels of 154 known genes were obviously altered, and these genes were involved in learning and memory, immune/inflammatory responses, apoptosis, response to stress, and signal transduction. The main results are discussed below.

Overproliferation of all glial cells is a universal event in many types of CNS damage. Glial cells are required for the development, formation and repair of neurons, and the axonal regeneration process is guided by these cells. In the present study, overproliferation of all glial cells caused by exposure to CeCl_3_ indicated that inflammatory/immune responses occurred in hippocampal tissue in addition to hippocampal injury. Secretoglobin, family 1A, member 1 (SCGB1A1) is the most studied member of the SCGB gene superfamily, its encoded product is a multifunctional protein with anti-inflammatory properties and a manifestation of anti-allergic, anti-chemotactic and anti-tumorigenic activity [31], [32]. Our data suggested that SCGB1A1 was significantly up-regulated with a Diffscore of 74.04 (Table S1), which may be associated with inflammatory/immune responses in the Ce^3+^-treated hippocampus. Adenosine a2B receptor (ADORA2B) is a member of the adenosine receptor group of G-protein-coupled receptors. ADORA2B plays a role in the relaxation of smooth muscle in the vasculature and intestines, inhibits monocyte and macrophage function and stimulates mast cell mediator release. Studies have shown that genetic deficiency of ADORA2B increased the death rate of mice suffering from cecal ligation and puncture-induced sepsis, and the increased mortality of ADORA2B knockout mice may be associated with increased levels of inflammatory cytokines, chemokines, augmented NF-κB and p38 activation in the spleen, heart, and plasma [33]. In the study by Frick et al., the endogenous protective molecule, ADORA2B, was expressed on intestinal epithelial cells [34]. In the current study, ADORA2B was down-regulated with a Diffscore of −16.41 (Table S1), which may promote inflammatory responses in the hippocampus following exposure to CeCl_3_. FCRLS belongs to a family which includes an intriguing group of cell surface receptors with preferential B cell expression. It has been shown to positively or negatively modulate the antibody-mediated responses of lymphocytes and inflammatory cells [35] and has important pathophysiologic roles in autoimmunity, allergy and inflammation [36]. Fc receptor-like s, scavenger receptor (FCRLS) deficient mice have profoundly altered humoral immune responses, immediate hypersensitivity, cytotoxic inflammatory responses and immune complex mediated inflammation [37], [38]. CeCl_3_ exposure led to significant down-regulation of FCRLS with a Diffscore of −68.11 (Table S1), which may also be related to inflammatory/immune responses in the Ce^3+^-treated hippocampus. In addition, guanine nucleotide binding protein, alpha q polypeptide (GNAQ), neurexin III (NRXN3) and rho/rac guanine nucleotide exchange factor (GEF) 2 (LBCL1) levels involved in the development, maturation, repair and regeneration of neurons were also significantly increased with Diffscores of 39.97, 29.42 and 28.26, respectively (Table S1). It is known that GNAQ transduces signals from the α_1_-adrenergic receptor to stimulate inositol-1,4,5-trisphosphate and diacylglycerol generation via phospholipase C, and then activates additional downstream effectors, to regulate a diverse range of biological functions. Mueller et al. indicated that as a strategy, increased GNAQ could improve neurite growth and sprouting after nerve damage [39]. NRXN3 is a cell adhesion molecule which helps to specify and stabilize synapses and provide receptors for neuroligins, neurexophilins, dystroglycans and a-latrotoxins [40]. It has been linked to many addictions such as cocaine, alcohol and morphine, suggesting that NRXN3 may play a crucial role in the synaptic plasticity of neurons in the basal ganglia, where they regulate reward-related learning [41]. LBCL1 and its negative regulator dynlt1, dynein light chain tctex-type 1d (Tctex-1) determine the genesis of neurons from precursors in the embryonic murine cortex [42]. In addition, Tctex-1 is selectively enriched in almost all cycling progenitors, young neuronal progeny, immature progenitors and migrating neuroblasts, but not in mature granular cells and astrocytes [43]. Increased LBCL1 may inhibit the differentiation, maturity and migration of neurons in mammalian brain. FBJ osteosarcoma oncogene (Fos) is a proto-oncogene. Its product dimerizes with members of the Jun family to form the transcription factor AP-1, which regulates a series of genes in response to many stimuli [44]. It has been proposed that Fos has a critical role in signal transduction, cell proliferation and differentiation [45]. Reports have demonstrated that the level of Fos expression was decreased in the LC (locus coeruleus) from rats treated acutely or chronically with morphine [46], and Fos knockout mice were growth-retarded, developed osteopetrosis with deficiencies in bone remodelling and tooth eruption, and have altered hematopoiesis [47]. In the present study, FOS gene was significantly down-regulated with a Diffscore of −19.89 (Table S1). Therefore, up-regulation of GNAQ, NRXN3 and LBCL1, and down-regulation of FOS by exposure to CeCl_3_ may result in inhibition of the development, maturation, repair and regeneration of neurons, and subsequently decreased spatial recognition memory in mice.

In the present study, our findings suggested that long-term exposure to low dose CeCl_3_ promoted ROS production (such as O_2_^−^ and H_2_O_2_) and led to peroxidation of lipids, proteins, and DNA (Table 3), which led to hippocampal apoptosis (Fig. 3). ROS are one of the triggers for intrinsic apoptosis. The overproduction of ROS has been shown to be closely associated with the induction of apoptotic and necrotic cell death in cell cultures [48]. This breaks down the balance of the oxidative/antioxidative system in the brain, resulting in lipid peroxidation, which increased the permeability of mitochondrial membrane [49]. In our previous studies, Ln^3+^ was also shown to mediate apoptosis in the spleen, liver in mice through the induction of ROS [13], [17]. However, the apoptotic mechanism in Ln^3+^-induced neurotoxicity remains unclear. In the present study, our data indicated that the expression of genes related to apoptosis, such as apoptosis antagonizing transcription factor (TRB), ubiquitin-conjugating enzyme e2 variant 1 (UBE2V1), csrnp1, cysteine-serine-rich nuclear protein 1 (AXUD1) and cell division cycle 37 homolog (CDC37), were significantly increased with Diffscores of 28.24, 41.69, 72.68 and 28.98 (Table S1), respectively. It was demonstrated that the protein encoded by TRB is involved in cell cycle control, gene transcription, and apoptotic signaling in neural tissues, therefore, TRB in cortical neurons exhibits anti-apoptotic activity, protecting cells from neuronal damage [50]. UBE2V1 is known to encode an ubiquitin conjugating enzyme variant. Syed identified UBE2V1 as a potential proto-oncogene, showing that high-level expression of UBE2V1 in cultured human cells caused a significant increase in NF-κB activity as well as the expression of Bcl-2, which is a target anti-apoptotic protein [51]. The up-regulation of UBE2V1 also conferred prolonged cell survival and protected cells against apoptosis induced by diverse stressors. AXUD1 is a member of a novel gene family encoding nuclear proteins which contain cysteine- and serine-rich domains, and is often considered to be related to reduced apoptosis [52]. CDC37 is an essential component of the mitogen-activated kinase protein (MAPK) signaling pathway. The protein encoded by CDC37 is thought to specifically strengthen the interaction between Hsp90 and kinase clients [53], which are involved in tumorigenesis, and interruption of Hsp90-managed pathways has a broad effect on cell growth and susceptibility to apoptosis [54]. It was demonstrated that CDC37 is required for G1 cell cycle progression, plays a critical role in v-Src oncogenesis and is required to maintain multiple protein kinase pathways implicated in apoptosis induction [55]. Therefore, brain apoptosis following exposure to CeCl_3_ may lead to upregulation of TRB, UBE2V1, AXUD1 and CDC37 expressions. Specifically, increased TRB, UBE2V1, and AXUD1 levels perhaps promoted anti-apoptotic activities, protecting cells from neuronal damage following Ce^3+^-induced neurotoxicity.

Previous studies have suggested that the reduction in learning and memory in rats or mice caused by La^3+^ and Ce^3+^ were related to significant increases in acetylcholine (Ach), glutamic acid (Glu), and nitric oxide (NO), and marked decreases in neurotransmitters such as norepinephrine (NE), 5-hydroxy tryptophan and its metabolite 5-hydroxy indole acetic acid, as well as dopamine and its metabolite 3, 4-dihydroxyphenylacetic acid [18], [22]. In addition, Ce^3+^ exposure resulted in a significant reduction in Ca^2+^ concentration in mouse brain [18]. Ln^3+^-induced neurotransmitter and Ca^2+^ changes were thought to be related to alterations in gene expressions in the brain [18]. In the present study, our data showed decreases in Slc5a7 and ADCY8 expression with Diffscores of −14.98, and −16.62, and an increase in DCAMKL1 expression with a Diffscore of 23.33 in the CeCl_3_-treated hippocampus (Table S1), respectively. Solute carrier family 5 (choline transporter), member (Slc5a7) is expressed in cholinergic neurons and is efficiently transported to axon terminals where it controls the rate-limiting step in acetylcholine synthesis [56]. Ferguson et al. demonstrated that Slc5a7 is an essential and regulated presynaptic component of cholinergic signaling and Slc5a7 warrants consideration as a candidate gene for disorders characterized by cholinergic hypofunction [57]. In the CNS, the cholinergic system plays an important role in learning and memory ability, and brain cholinergic dysfunction results in dementia with symptoms such as memory loss and disorientation in cerebrovascular or Alzheimer’s disease [58]. Adenylate cyclase 8 (ADCY8 or AC8) is a pure Ca^2+^ sensor, catalyzing the transformation of ATP to cAMP, with an important role in neuronal plasticity. The deletion of ADCY8 can exacerbate neuroapoptosis in mice exposed to ethanol [59]. The AC8 knockout mice exhibited mossy fiber long-term potentiation (LTP) defects comparable with wild type mice, and short-term plasticity was also disrupted [60]. All these reports provided us with credible evidence that the decrease in Ca following Ce^3+^ exposure was related to down-regulation of ADCY8 expression, which in turn, exacerbated neuroapoptosis and disrupted mossy fiber LTP. Decreased Slc5a7 and Adcy8 expression due to CeCl_3_ exposure may be related to overproduction of Ach, Ca reduction, and subsequent mental retardation. The doublecortin-like kinase 1 (DCAMKL1) gene encodes a member of the protein kinase superfamily and the doublecortin family. The protein encoded by DCAMKL1 has microtubule-polymerizing activity and is involved in several different cellular processes, including neuronal migration, retrograde transport, neuronal apoptosis and neurogenesis. The DCAMKL1 gene can be up-regulated by brain-derived neurotrophic factor and is associated with memory and general cognitive abilities. Transgenic mice with over-expression of brain CaMK Related Peptide (CARP) were shown to have decreased hippocampal CA3/CA1 network excitability. Schenk et al proposed that the DCAMKL1 gene product affects glutamatergic neuronal transmission in response to neurological stimuli [61, 62]. Therefore, the decrease in learning and memory ability, and Glu overaccumulation induced by Ln^3+^ may be associated with increased DCAMKL1 expression.

### Conclusion

The present study suggests that long-term exposure to CeCl_3_ at 0.5, 1, and 2 mg/kg dose resulted in hippocampal damage, oxidative stress, and a decrease in spatial recognition memory. Furthermore, hippocampal dysfunction following exposure to CeCl_3_ may be closely related to significant changes in the expression of genes involved in learning and memory, apoptosis, response to stress, immunity and inflammation, and signal transduction. Considering the average intake of Ln (1.75–2.25 mg/day) in humans, the application of cerium in crop production, animal breeding, and medicine should be carried out cautiously.

## Supporting Information

Table S1 Genes of known function were significantly altered after intragastric administration of 2 mg/kg BW CeCl_3_ for 90 consecutive days.
(DOC)
